RETRACTED

# MiRNA-200b Regulates RMP7-Induced Increases in Blood-Tumor Barrier Permeability by Targeting RhoA and ROCKII

**DOI:** 10.3389/fnmol.2016.00009

**Published:** 2016-02-05

**Authors:** Teng Ma, Yi-xue Xue

**Affiliations:** ^1^Department of Neurobiology, College of Basic Medicine, China Medical UniversityShenyang, China; ^2^Institute of Pathology and Pathophysiology, China Medical UniversityShenyang, China

**Keywords:** microarray, miR-200b, RMP7, RhoA, ROCKII, BTB

## Abstract

The primary goals of this study were to investigate the potential roles of miR-200b in regulating RMP7-induced increases in blood-tumor barrier (BTB) permeability and some of the possible molecular mechanisms associated with this effect. Microarray analysis revealed 34 significantly deregulated miRNAs including miR-200b in the BTB as induced by RMP7 and 8 significantly up-regulated miRNAs in the BTB by RMP7. RMP7 induced tight junction (TJ) opening of the BTB, thereby increasing BTB permeability. Associated with this effect of RMP7 was a decrease in miR-200b expression within the human cerebral microvascular endothelial cells line hCMEC/D3 (ECs) of the BTB. Overexpression of miR-200b inhibited endothelial leakage and restored normal transendothelial electric resistance values. A simultaneous shift in occludin and claudin-5 distributions from insoluble to soluble fractions were observed to be significantly reduced. In addition, overexpression of miR-200b inhibited the relocation of occludin and claudin-5 from cellular borders into the cytoplasm as well as the production of stress fiber formation in GECs (ECs with U87 glioma cells co-culturing) of the BTB. MiR-200b silencing produced opposite results as that obtained from that of the miR-200b overexpression group. Overexpression of miR-200b was also associated with a down-regulation in RhoA and ROCKII expression, concomitant with a decrease in BTB permeability. Again, results which were opposite to that obtained with the miR-200b silencing group. We further found that miR-200b regulated BTB permeability by directly targeting RhoA and ROCKII. Collectively, these results suggest that miR-200b's contribution to the RMP7-induced increase in BTB permeability was associated with stress fiber formation and TJ disassembly as achieved by directly targeting RhoA and ROCKII.

## Introduction

RMP7, a synthetic bradykinin (BK) analog, is a potent and specific BK B2 receptor agonist. RMP7 has a longer plasma half-life and less toxicity than BK and can selectively bind to B2 receptors on endothelial cells thus forming a tight junction (TJ) (Bartus et al., 1996). The interaction of BK or RMP7 with the B2 receptor results in a rapid, but transient, increase in the permeability of the blood-brain barrier (BBB) and blood-tumor barrier (BTB) (Inamura et al., 1994; Elliott et al., 1996; Matsukado et al., 1996; Bartus et al., 2000; Emerich et al., 2000). It has been reported that intracarotid infusion of RMP-7 is shown to increase the delivery of carboplatin more than 2-fold and to improve survival in a rat glioma model (Emerich et al., 1999). In line with these findings, the results from our laboratory demonstrated that BK increased the permeability of the BTB (Ma and Xue, 2010; Ma et al., 2012).

RETRACTED

MicroRNAs (miRNAs) are non-coding, single-stranded, small RNA molecules of approximately 20–22 nucleotides in length that can inhibit gene expression at the post-transcriptional level through nucleotide base pairings between complementary sequences of miRNAs and the 3′ untranslated regions (3′-UTR) (Wei and Pei, 2010; Wang et al., 2012). MiRNAs have been shown to play important roles in embryonic development, cancer, as well as in a variety of other physiological and pathological processes (Alvarez-Garcia and Miska, 2005). The paucity of data on miRNA alterations during the process of RMP7-induced TJ opening of the BTB and the implications for the potential use of miRNAs as biomarkers in therapeutic approaches led us to evaluate the differential expression of miRNAs by microarray analysis and quantitative real-time PCR (Quantitative RT-PCR) in response to RMP7.

The small GTPase, RhoA, and its downstream effector, ROCKII, the major downstream effector of activated RhoA, are known to stimulate F-actin rearrangement and regulate a number of cellular processes, including cytoskeletal dynamics, cell polarity, membrane transport, and gene expression (Jaffe and Hall, 2005; Bryan et al., 2010). In addition, RhoA/ROCKII signaling is believed to serve as an important signal molecule which contributes to stress fiber formation as associated with TJ disassembly and increased endothelial permeability (Wojciak-Stothard et al., 2006; Chen et al., 2011; Han et al., 2013; Mangialardi et al., 2013). In accord with these reported actions of RhoA/ROCKII signaling are the results from our laboratory which demonstrate that RhoA/ROCKII signaling was required for a BK-induced increase in BTB permeability (Ma and Xue, 2010; Ma et al., 2012). However, the underlying mechanisms remain unclear. Results from recent studies have revealed that miR-133b promotes neurite outgrowth and miR-122 suppresses hepatocellular carcinoma cell motility and invasion by targeting RhoA (Wang et al., 2014a; Lu et al., 2015). As indicated by gene ontology analysis, a predominant effect of miR-200b targets involve that of a widespread, coordinated control of actin cytoskeleton dynamics. Functional characterizations of these miR-200b targets indicate that they constitute sub-networks that underlie the ability of cancer cells to migrate and invade, including the coordination of effects on Rho-ROCK signaling, cytoskeletal remodeling, invadopodia formation and MMP activity (Bracken et al., 2014). These studies demonstrate that miR-200b and other miRNAs could regulate the Rho-ROCK signal pathway by directly targeting RhoA and ROCK.

RETRACTED

The primary goals of this study were to, (1) identify critical miRNAs associated with RMP7-induced TJ opening of the BTB and (2) perform a comprehensive analysis of miRNA regulation in RhoA and ROCKII expression in GECs (ECs with U87 glioma cells co-culturing) of the BTB. To accomplish these goals, the regulatory effects of potential miRNAs on RhoA and ROCKII were investigated along with the potential mechanisms of RMP7-induced TJ opening in the BTB.

## Materials and methods

### Cell lines and cultures

The immortalized human cerebral microvascular endothelial cell line hCMEC/D3 (ECs) was a generous gift from Dr. Couraud (Institut Cochin, Paris, France). The cells were cultured on culture flasks coated with 150 mg/ml of cultrex rat collagen I (R&D Systems, Minneapolis, MN) in EBM-2 medium (Lonza, Walkersville, MD, USA, Paisley, UK) containing 1% chemically defined lipid concentrate (Life Technologies Corporation, Paisley, UK), 5 mg/ml ascorbic acid (Sigma–Aldrich, St Louis, MO, USA) and 1 ng/ml human basic fibroblast growth factor (bFGF, Sigma–Aldrich), supplemented with 5% fetal bovine serum (FBS, PAA Laboratories GmbH, Pasching, Austria). The ECs were cultured at 37°C in a humidified atmosphere containing 5% CO_2_, and cells at passages 30–40 were used for the experiments, with medium being refreshed every 3–4 days.

The U87 human glioblastoma cell line was obtained from the Shanghai Institute for Biological Sciences Cell Resource Center. The cells were cultured in Dulbecco's modified Eagle's medium (DMEM) with high glucose and 10% fetal bovine serum in a humidified atmosphere of 5% CO_2_ at 37°C.

### The *in vitro* BTB model

To establish *in vitro* BTB models, U87 cells were seeded at 2 × 10^4^ per well in six-well plates and cultured for 2 days. After the U87 cells were confluent, ECs were seeded at 2 × 10^5^ per well in the upper compartment of the transwell system (0.4 mm pore size; Corning, NY). ECs and U87 cells were co-cultured in the transwell system for 4 days according to procedures previously established within our laboratory (Ma and Xue, 2010; Ma et al., 2012, 2014a; Zhao et al., 2015). These co-cultured endothelial cells were referred to as glioma endothelial cells (GECs) as compared with that of the ECs.

RETRACTED

### MiRNA expression profiles and MiRNA target analyses

A total of 10 samples from 2 different groups were used in this study. The 2 basic groups from which these samples consisted of the BTB control group (ECs monolayer, with U87 glioma cells co-culturing) and the RMP7 group, with 10 min durations of RMP7 exposure. Total RNA from GECs was collected with use of the Qiagen miRNeasy Mini kit (Qiagen Inc., Germantown, MD, USA) according to the manufacturer's instructions. MiRNA expression profiles were performed using the TaqMan MicroRNA Assay Human Set (Applied Biosystems, Foster, VA, USA) on the 7900HT Fast Real-Time PCR System (Applied BIosystem, Foster City, CA, USA), according to the manufacturer's instructions. Raw cycle threshold (Ct) values were calculated using SDS 2.3 and RQ manager 1.2 software (Applied Biosystems) as achieved by applying automatic baseline and threshold settings. RNU-44 was used as an endogenous control. The –ΔCt was calculated and heatmap analysis was performed with hierarchical clustering. Target prediction was performed using the open source program miRTarBase, MiRDB, Targetscan, Miranda and Pictar (http://mirtarbase.mbc.nctu.edu.tw/, http://www.mirdb.org/miRDB/, http://www.targetscan.org/, http://www.microrna.org/ and http://pictar.mdc-berlin.de/).

### Drug treatment and experimental groups

RMP7 (5 nmol/l Sigma–Aldrich, St Louis, MO, USA) was added to the upper chamber (Prados et al., 2003; Packer et al., 2005). There were seven groups in our present study (*n* = 5/group): the control group (BTB group, ECs monolayer with U87 glioma cells co-culturing) and 6 RMP7 groups consisting of RMP7 exposure for 0, 5, 10, 15, 30, or 60 min.

### Measurement of transendothelial electric resistance (TEER)

The electrical resistance of GEC monolayers cultured on transwell filters was measured using a Millicell-ERS instrument (Millipore, Billerica, MA, USA). Electrical resistance was expressed in units of Ω cm^2^ using the surface area of the transwell insert (Ma and Xue, 2010; Ma et al., 2012, 2014a; Zhao et al., 2015).

### Horseradish peroxidase (HRP) flux measurement

Horseradish peroxidase (HRP, Sigma-Aldrich) at 0.5μmol/l in serum-free EBM-2 was added to the upper chamber of the transwell system after *in vitro* BTB models were successfully established. Following RMP7 administration at the times indicated, the media from the lower chamber was collected. The HRP flux was expressed as picomoles passed per cm^2^ surface area (Ma and Xue, 2010; Ma et al., 2012, 2014a; Zhao et al., 2015).

### Reverse transcription and quantitative real time PCR (quantitative RT-PCR)

This assay was used to detect mRNA expression levels of miR-200b in GECs, the efficiency of miR-200b transfection and mRNA expression levels of RhoA and ROCKII in GECs of the BTB. MiRNAs were extracted with use of a miRNA Isolation Kit (RNAiso for Small RNA, TaKaRa, Dalian, China) according to the manufacturer's instructions. Total RNAs were isolated using Trizol reagent (Life Technologies Corporation, Carlsbad, CA, USA) according to the manufacturer's instructions. Reverse transcription was performed with use of a PrimeScriptTM RT reagent Kit (TaKaRa, Dalian, China) according to the manufacturer's instructions. Quantitative RT-PCR was performed with use of a PCR kit (TaKaRa, Dalian, China). Quantitative RT-PCR primers for mir-200b (DHM0179) and U6 (D356-03) were purchased from TaKaRa (TaKaRa, Dalian, China). The forward and reverse primers of each PCR set, the sizes of PCR products, GenBank accession numbers, oligonucleotides, and annealing temperatures are presented in Table 1. PCR was performed for forty cycles with the following parameters: 10 s at 95°C, and for each cycle 5 s at 95°C for denaturing and 20 s at 60°C for annealing. All quantitative RT-PCR analyses were conducted with use of a 7500 Fast Real-Time PCR System (Applied Biosystems). Expression levels of miR-200b and other genes were normalized to that of the U6 housekeeping gene and GAPDH by the delta Ct value, respectively.

RETRACTED

**Table 1:** **Oligonucleotides used for quantitative RT-PCR, their Amplicon Size, GenBank accession number, and annealing temperatures**.

**Gnen**	**Sequence**	**Amplicon size**	**Genbank accession number**	**Annealing Temperature**
RhoA	(F) 5′-TCTGTCCCAACGTGCCCATC -3′ (R) 5′-CCCAAAAGCGCCAATCCTGT -3′	149	NM_001664.2	60°C
ROCKII	(F) 5′-CTCCATTTTATGCGGATTCACTTG-3′ (R) 5′-TGATTTCTTCCACCCCATTTCTC-3′	171	NM_004850.3	60°C
GAPDH	(F)5′-AAATCCCATCACCATCTTCCAG -3′ (R) 5′-TGATGACCCTTTTGGCTCCC -3′	149	NM_002046.4	60°C

### Cell transfection

The miRNA-200b mimics (GenePharma, Shanghai, China), miRNA-200b inhibitors (GenePharma, Shanghai, China) and their negative control molecules were synthesized by GenePharma. The sequence of miRNA-200b mimic and inhibitor were as follows: UAAUACUGCCUGGUAAUGAUGAAUCAUUACCAGGCAGUAUUAUU and UCAUCAUUACC AGGCAGUAUUA, respectively. The sequence of their corresponding negative control molecules were as follows: UUCUCCGAACGUGUCACGUTTACGUGACACGUUCGG AGAATT and CAGUACUUUUGUGUAGUACAA, respectively. GECs at 60–80% confluence in the upper compartment of transwell inserts were transfected with oligonucleotides using lipofectamine 3000 reagent (Life Technologies Corporation, Carlsbad, CA, USA) according to the manufacturer's instructions and were added directly to the cells to a final oligonucleotide concentration of 50 nM. After transfection for 72 h, the medium was replaced with fresh EBM-2 medium containing 5% fetal bovine serum and the cells were incubated for 96 h. The transfected efficacy of miRNA-200b mimics and miRNA-200b inhibitors were analyzed by real-time PCR. Those transfected with miRNA precursors were divided into 5 groups: (1) controls with no miRNA precursor but containing PBS, (2) pre-miR-con containing a pre-miR negative control precursor, (3) pre-miR-200b containing a miR-200b precursor, (4) anti-miR-con containing an anti-miR negative control precursor, and (5) anti-miR-200b containing a miR-200b inhibitor precursor.

RETRACTED

### Cell fractionation and western blot

Confluent GECs were washed three times with Dulbecco's phosphate-buffered saline (D-PBS) containing 0.1 mM ethylenediamine tetraacetic acid (EDTA) without calcium and magnesium. The GECs were homogenized in 1 ml lysis buffer A [2 mM EDTA, 10 mM ethylene glycol tetraacetic acid (EGTA), 0.4% NaF, 20 mM Tris-HCl, protease inhibitor cocktail, 1% Triton X-100, pH 7.5] at 4°C. Samples were centrifuged at 14,000 g for 30 min, the supernatant was transferred to a separate tube and collected as the soluble fraction (S). Buffer A (150 μl) with 1% sodium dodecyl sulfate (SDS) at 4°C was then added to the pellet. The pellet was disrupted with an ultrasonic crusher. Samples were then centrifuged at 14,000 g for 30 min at 4°C as described above. The supernatant was collected as the insoluble fraction (IS). Equal amounts of proteins (40–50 μg) were separated and processed for immunoblotting with antibodies for claudin-5 (diluted1:250; Life Technologies Corporation, Frederick, MD, USA), occludin (diluted 1:250; Life Technologies Corporation, Frederick, MD, USA), RhoA (diluted 1:300; Abcam, Cambridge, UK) and ROCK II (diluted 1:300; geneTex, Irvine, California, USA). All protein bands were scanned using ChemiImager 5500 V2.03 software. The integrated density values (IDV) were calculated by computerized image analysis system (Fluor Chen 2.0) and normalized with that of GAPDH.

### Immunofluorescence

U87 cells were trypsinized, then plated onto 6-well culture plates with suitable culture medium (high-glucose DMEM, 10% fetal bovine serum, 100 U/ml penicillin, 100 μg/ml streptomycin) containing 10^3^ cells. When 80% of the U87 cells were confluent, the complete culture media was aspirated and replaced with fresh EBM-2 medium containing 5% fetal bovine serum. EC monolayers grown on glass coverslips were placed into culture plates and co-cultured for 4 days. The GEC monolayers grown on glass coverslips were fixed with 4% paraformaldehyde and permeabilized with 0.5% Triton X-100. After blocking with 2% bovine serum albumin (BSA) in PBS, the cells were incubated with mouse anti-occludin (diluted 1:50; Life Technologies Corporation, Frederick, MD, USA) and rabbit anti-claudin-5 (diluted 1:50; Life Technologies Corporation, Frederick, MD, USA) to visualize the distribution of occludin and claudin-5, respectively. The cells were incubated with rhodamine-labeled phalloidin (diluted 1:250; Sigma-Aldrich) to assess actin filaments. The cells were incubated with mouse anti-RhoA (diluted 1:150; Abcam, Cambridge, UK) and rabbit anti-ROCK II (diluted 1:50; GeneTex, Irvine, California, USA) to analyze their expression. The glass slides were then evaluated using immunofluorescence microscopy (Olympus, Japan).

RETRACTED

### Plasmid construction and dual-luciferase reporter assay

The target genes of miR-200b were predicted with the help of Bioinformatics software: miRTarBase, MiRDB, Targetscan, Miranda and Pictar (http://mirtarbase.mbc.nctu.edu.tw/, http://www.mirdb.org/miRDB/, http://www.targetscan.org/, http://www.microrna.org/ and http://pictar.mdc-berlin.de/). Wild-type RhoA and ROCKII 3′-UTR reporter plasmids (RhoA wt and ROCKII wt) and mutated-type RhoA and ROCKII 3′-UTR reporter plasmids (RhoA mut and ROCKII mut) were cloned to pmirGLO-promoter vector according to the miR-200b seed sequence (GenePharma, Shanghai, China). A plasmid carrying a non-targeting sequence was used as a negative control (NC). HEK 293 T cells were seeded and cultured in 96-well microtiter plates (Corning, NY) for 24 h. HEK 293 T cells were then transfected with the pmirGLO empty vector (marked as “Control”), co-transfected with the wild-type or mutated RhoA and ROCKII 3′-UTR reporter plasmids or transfected with pre-miR-200b or pre-miR-con precursors. Luciferase assays were performed 48 h after transfection using the Dual-Luciferase Reporter Assay System (Promega, WI, USA).

### Data analysis

Experiments were replicated a minimum of three times. Data are presented as means ± standard deviations (SD). Comparisons among more than two groups were performed using a one-way analysis of variance (ANOVA) followed by Dunnett's test for *pos-hoc* comparisons. A *P* < 0.05 was required for results to be considered statistically significant.

## Results

### Effect of RMP7 on changes in distinct MiRNA expression profiles in the BTB

MiRNA gene expression profiles were successfully obtained from samples in each group. In total, 322 miRNAs were detected in the TaqMan® Array MicroRNA human card A and B (Figure 1A and see Supplementary Material). Heat-map analysis was performed using the -ΔCT value and showed that the expression of most miRNAs appeared quite consistent across the different samples, indicating that the overall miRNA gene expression profiles among different individuals were consistent. A -ΔCT value > 35 was established as a cut off and was then not subjected to further analysis. Microarray analysis revealed 34 significantly deregulated miRNAs including miR-200b in the BTB as induced by RMP7 and 8 significantly up-regulated miRNAs in the BTB by RMP7 as compared with that observed within the BTB control (Figure 1B). After being treated with RMP7, the expression of miR-200b was significantly down-regulated by 3.3 ± 0.6-fold as compared with that of the BTB control group (Figure 1B). This reduction in miR-200b expression ranked third when considering all deceased miRNAs as determined by gene chip.

RETRACTED

**Figure 1:** **Effect of RMP7 on changes in distinct miRNA expression profiles of the BTB. (A)** MiRNA gene expression profiles as obtained from samples in the BTB and RMP7 groups. **(B)** miRNA expression in RMP7 10 min group was significantly up-regulated and down-regulated compared to BTB group.

Conserved sequences are similar or identical with those that occur within nucleic acid sequences (such as RNA and DNA sequences). In the case of cross species conservation, this indicates that a particular sequence may have been maintained by evolution, despite speciation. Conserved sequences in the 3′-UTR of RhoA and ROCKII are CAGUAUU and ACUAUUA, respectively. Validated target genes were analyzed using the databases of miRTarBase, MiRDB, Miranda, TargetScan and Pictar repositories. As based upon the results of these analyses, binding of miRNA-200b to both RhoA and ROCKII was observed using MiRDB, Miranda and TargetScan, while use of miRTarBase indicated that binding of miRNA-200b was observed only to ROCKII, and Pictar indicated an absence of miRNA-200b binding to either RhoA or ROCKII. Moreover, miR-200b was shown to have a putative binding site at the 3′-UTR region of RhoA and ROCKII with a 100% conserved sequence as revealed by TargetScan (data not shown).

### RMP7 decreased the expression of MiR-200b in GECs

As shown in Figure 2, RMP7 significantly induced a time dependent decrease in miR-200b mRNA expression, with nadir values being obtained at 10 min after RMP7 treatment. Thereafter, miR-200b expressions gradually increased and were restored to their original basal levels.

**Figure 2:** **Relative expression of miR-200b as detected by quantitative RT-PCR**. GECs from the RMP7 groups were treated with RMP7 (5 nmol/l) for 0, 5, 10, 15, 30, or 60 min. U6 RNA level was used as an internal control. Values are means ± SD (*n* = 5/group). ^*^P < 0.05 vs. the other groups; *ns*, non-significant.

### Effect of RMP7 on changes in HRP flux and TEER of the BTB

GECs from the RMP7 groups were treated with RMP7 (5 nmol/l) for 0, 5, 10, 15, 30, or 60 min. After RMP7 administration, TEER values were decreased by 5 min, reaching their lowest values at 15 min and increased thereafter (Figure 3A). Meanwhile, we observed that RMP7 significantly increased HRP flux in a time-dependent manner, with peak levels observed at 15 min after RMP7 treatment (Figure 3B). These results, as obtained with the TEER and HRP flux assays, revealed that the TJ of the BTB was opened by RMP7; results which were consistent with our previous findings demonstrating a BK-induced TJ opening of the BTB (Liu et al., 2008; Ma and Xue, 2010; Ma et al., 2012).

RETRACTED

**Figure 3:** **Effect of RMP7 on changes in HRP flux and TEER of BTB. (A)** TEER values of GECs were expressed as Ω cm^2^. GECs from RMP7 groups were treated with RMP7 (5 nmol/l) for 0, 5, 10, 15, 30, or 60 min. Values are means ± SD (*n* = 5/group). ^*^P < 0.05 vs. control group; ^#^*P* < 0.05 vs. the other groups. **(B)** HRP flux was calculated as pmol/cm^2^. GECs from the RMP7 groups were treated with RMP7 (5 nmol/l) for 0, 5, 10, 15, 30, or 60 min. Values are means ± SD (*n* = 5/group). ^*^P < 0.05 vs. control group; ^#^*P* < 0.05 vs. the other groups.

### Verification of transfected efficiency for MiR-200b mimics and inhibitors

Quantitative RT-PCR was performed to detect the transfected efficacy of miRNA-200b mimics and miRNA-200b inhibitors. As shown in Figure 4, a time-dependent increase of miRNA-200b expression in the pre-miR-200b group was observed, with maximal miRNA-200b expression occurring at 72 h. The expression of miR-200b in the pre-miR-200b group was significantly up-regulated by 6.862 ± 0.725 and 6.819 ± 0.838-fold as compared with that of the control and pre-miR-con groups, respectively (Figure 4). Following miRNA-200b inhibitor transfection, a time-dependent decrease of miR-200b expression was observed, with nadir levels obtained at 72 h, and the expression of miR-200b increasing thereafter (Figure 4). The expression of miR-200b in the anti-miR-200b group was significantly down-regulated by 0.210 ± 0.027 and 0.207 ± 0.027-fold as compared with that of the control and anti-miR-con groups, respectively (Figure 4). Maximal transfection efficacy of the oligonucleotides both occurred at 72 h. Therefore, the time period of 96 h after transfection was considered as the best time for harvest and use in the subsequent experiments.

**Figure 4:** **Transfection efficiency for miR-200b mimics and inhibitors as detected by quantitative RT-PCR**. MiR-200b mimics and inhibitors were transfected into GECs. U6 RNA level was used as an endogenous control. Values are means ± SD (*n* = 5/group). ^*^P < 0.05 vs. control group; ^#^*P* < 0.05 vs. NC group; ^▵^*P* < 0.05 vs. the other groups.

RETRACTED

### Overexpression or silencing of MiR-200b significantly changed the integrity and permeability of BTB

TEER values in the pre-miR-200b group were significantly increased as compared with the control and pre-miR-con groups; while TEER values in the anti-miR-200b group were markedly decreased as compared with the control and anti-miR-con groups (Figure 5A). No statistically significant differences were present among the control, pre-miR-con and anti-miR-con groups (Figure 5A). HRP flux in the pre-miR-200b group was significantly decreased as compared with the control and pre-miR-con groups; whereas HRP flux in the anti-miR-200b group was dramatically increased as compared with the control and anti-miR-con groups (Figure 5B). No significant differences were obtained among the control, pre-miR-con and anti-miR-con groups (Figure 5B).

**Figure 5:** **Changes in BTB integrity and permeability after overexpression or silencing of miR-200b. (A)** TEER values of GECs expressed as Ω cm^2^. Values are means ± SD (n = 5/group). ^*^P < 0.05 vs. control group; ^#^*P* < 0.05 vs. pre-miR-con group; ^▵^*P* < 0.05 vs. anti-miR-con group;^▿^*P* < 0.05 vs. pre-miR-200b group. **(B)** HRP flux was calculated as pmol/cm^2^. Values are means ± SD (*n* = 5/group). ^*^P < 0.05 vs. control group; ^#^*P* < 0.05 vs. pre-miR-con group; ^▵^*P* < 0.05 vs. anti-miR-con group;^▿^*P* < 0.05 vs. pre-miR-200b group.

### Overexpression or silencing of MiR-200b significantly changed a shift from insoluble to soluble fractions in occludin and claudin-5 distribution

Soluble fragments (S) of occludin and claudin-5 represent dephosphorylated forms of fragments and are susceptible to non-ionic detergent extraction. Insoluble fragments (IS) of occludin and claudin-5 represent phosphorylated forms of fragments, which combine with actin microfilaments through zonula occludens (ZOs) and are resistant to non-ionic detergent extraction (Li et al., 2006; Ma and Xue, 2010; Ma et al., 2012). As shown in Figure 6, a clear shift from insoluble to soluble fractions of occludin and claudin-5 distribution was observed in the pre-miR-200b and anti-miR-200b groups as revealed by Western-blot. Significant increases in the shifts of occludin and claudin-5 distribution were observed in the pre-miR-200b group as compared with the control and pre-miR-con groups; whereas a markedly decreased shift of occludin and claudin-5 distribution in the anti-miR-200b group was obtained as compared with the control and anti-miR-con groups. No statistically significant differences were present among the control, pre-miR-con and anti-miR-con groups.

RETRACTED

**Figure 6:** **IDV ratio of IS and S in occludin and claudin-5 as detected by Western blot after overexpression or silencing of miR-200b**. Soluble fragments (S) of occludin and claudin-5 represent dephosphorylated forms and are susceptible to non-ionic detergent extraction. Insoluble fragments (IS) of occludin and claudin-5 represent phosphorylated forms, which combine with actin microfilaments through zonula occludens (ZOs) and are resistant to non-ionic detergent extraction. Values are means ± SD (*n* = 5/group). ^*^P < 0.05 vs. control group; ^#^*P* < 0.05 vs. pre-miR-con group; ^▵^*P* < 0.05 vs. anti-miR-con group; ^▿^*P* < 0.05 vs. pre-miR-200b group.

### Effects of MiR-200b on relocation of occludin and claudin-5 and formation of stress fibers

F-actin was found to be localized mainly at the cell periphery (Figures 7K,L,N), where occludin and claudin-5, the two major components of TJs, are also localized (Figures 7A,B,D,F,G,I). Anti-miR-200b induced the formation of stress fibers within the center of the cell (Figure 7O), which was accompanied by a redistribution of occludin and claudin-5 from cellular membranes to the cytoplasm and nucleus (Figures 7E,J). Pre-miR-200b reduced the number of central stress fibers and strongly enhanced cell localization of F-actin within the periphery of GECs in the BTB (Figure 7M). Furthermore, pre-miR-200b decreased the redistribution of occludin and claudin-5 from cellular membranes to the cytoplasm and nucleus while enhancing cellular membrane localization of occludin and claudin-5 in GECs of the BTB (Figures 7C,H).

**Figure 7:** **Immunofluorescence analysis of occludin, claudin-5 and F-actin in GECs after overexpression or silencing of miR-200b**. **(A,B,D)** Each represents a control group, mimic negative control group, and inhibitor negative control group in occludin. **(F,G,I)** Each represents a control group, mimic negative control group, and inhibitor negative control group in claudin-5. **(K,L,N)** Each represents a control group, mimic negative control group, and inhibitor negative control group in F-actin. Anti-miR-200b induced formation of stress fibers in the center of the cell **(O)** and is accompanied by a redistribution of occludin and claudin-5 from cellular membranes to the cytoplasm and nucleus **(E,J)**. Pre-miR-200b reduced the number of central stress fibers and strongly enhanced cell peripheral localization of F-actin in GECs of the BTB **(M)**. Furthermore, pre-miR-200b decreased the redistribution of occludin and claudin-5 from cellular membranes to the cytoplasm and nucleus and enhanced cellular membrane localization of occludin and claudin-5 in GECs of the BTB **(C,H)**. Black arrows show the localization of peri-cellular dense aggregates of actin filaments in GECs. Green arrows show stress fibers. Scale bars represent 20 μm.

RETRACTED

### Effect of RMP7 on expression of RhoA and ROCKII in GECs of BTB

The mRNA and protein expression levels of RhoA and ROCKII were analyzed by real-time PCR and western blotting, respectively. As shown in Figure 8, mRNA and protein expressions of RhoA and ROCKII were increased after RMP7 administration. This RMP7-induced increase was time-dependent with maximum expression occurring at 10 min. Thereafter, mRNA and protein expressions of RhoA and ROCKII gradually returned to basal levels.

**Figure 8:** **Effect of RMP7 on expression of RhoA and ROCKII in GECs of the BTB**. GECs from RMP7 groups were treated with RMP7 (5 nmol/l) for 0, 5, 10, 15, 30, or 60 min. **(A)** Relative mRNA expressions of RhoA and ROCKII as determined by quantitative RT-PCR. GAPDH RNA levels were used as an endogenous control. Values are means ± SD (*n* = 5/group). ^*^P < 0.05 vs. control group; ^#^*P* < 0.05 vs. RMP7 0 min group;^▵^*P* < 0.05 vs. RMP7 15 min. **(B,C)** Protein expressions of RhoA and ROCKII as assessed with Western blot. Values are means ± SD (*n* = 5/group). ^*^P < 0.05 vs. control group; ^#^*P* < 0.05 vs. RMP7 0 min group;^▵^*P* < 0.05 vs. RMP7 15 min.

### Overexpression or silencing of MiR-200b regulates the expression of RhoA and ROCKII

As shown in Figure 9, both mRNA and protein expressions of RhoA and ROCKII were decreased in the pre-miR-200b group as compared with the control and pre-miR-con groups, but increased in the anti-miR-200b group as compared with the control and anti-miR-con groups. No statistically significant differences were obtained among the control, pre-miR-con and anti-miR-con groups (Figures 9A–C). Immunofluorescence analysis revealed that RhoA and ROCKII were mainly distributed in the cytoplasm and nuclei of GECs in the BTB (Figures 9D,E), with similar changes being observed in the alteration of mRNA and protein. An inverse relationship was present between the miR-200b and expressions of RhoA and ROCKII.

**Figure 9:** **Alteration of RhoA and ROCKII in GECs of the BTB after overexpression or silencing of miR-200b. (A)** Relative mRNA expressions of RhoA and ROCKII as determined by quantitative RT-PCR. GAPDH RNA levels were used as an endogenous control. Values are means ± SD (*n* = 5/group). ^*^P < 0.05 vs. control group; ^#^*P* < 0.05 vs. pre-miR-con group; ^▵^*P* < 0.05 vs. anti-miR-con group;^▿^*P* < 0.05 vs. pre-miR-200b group. **(B,C)** Protein expressions of RhoA and ROCKII as assessed with Western blot. Values are means ± SD (*n* = 5/group). ^*^P < 0.05 vs. control group; ^#^*P* < 0.05 vs. pre-miR-con group; ^▵^*P* < 0.05 vs. anti-miR-con group;^▿^*P* < 0.05 vs. pre-miR-200b group. **(D,E)** Distribution and expression of RhoA and ROCKII as detected with immunofluorescence assay. RhoA (green) and ROCKII (green) were, respectively, labeled with fluorescent secondary antibody and nuclei (blue) were labeled with DAPI. Scale bars represent 20 μm.

RETRACTED

### RhoA and ROCKII were direct targets of MiR-200b

Bioinformatics software (http://www.targetscan.org/) available on the public miRNA databases were used to predict a binding site between the seed region of miR-200b and 3′-UTR of RhoA and ROCKII. MiR-200b was shown to have a putative binding site to the 3′-UTR region of RhoA and ROCKII with a 100% conserved sequence. RhoA and ROCKII were predicted to harbor one highly conservative miR-200b binding site in the 3′-UTR at position 133–139 and 912–918, respectively. The seed for miR-200b to RhoA and ROCKII 3′-UTR is shown in Figures 10A,C. In order to assess whether RhoA and ROCKII were functional targets of miR-200b, luciferase reporter plasmids containing the wild-type 3′-UTR of RhoA and ROCKII (RhoA-3′UTR-Wt and ROCKII-3′UTR-Wt) were constructed. As expected, the relative luciferase activity of the RhoAwt.pre-miR-200b and ROCKII wt.pre-miR-200b groups were significantly decreased in comparison with that of the RhoAwt.pre-miR-con and ROCKII wt.pre-miR-con groups (Figures 10B,D). These results suggest that miR-200b inhibited the 3′-UTR function of RhoA and ROCKII. To further verify whether miR-200b directly targeted RhoA and ROCKII through the predicted binding site, luciferase reporter plasmids containing the Mut-type 3′-UTR of RhoA and ROCKII (RhoA-3′UTR-Mut and ROCKII-3′UTR-Mut) were constructed. Co-transfection of miR-200b and RhoA-3′UTR-Mut or ROCKII-3′UTR-Mut did not change luciferase activity (Figures 10B,D). These results indicate that RhoA and ROCKII were direct targets of miR-200b with the specific binding site being located at the seed sequence.

**Figure 10:** **MiR-200b inhibits the expression of RhoA and ROCKII by targeting their 3′-UTR. (A,B)** Putative binding sites of RhoA 3′-UTR and ROCKII 3′-UTR as matching with the seed region of miR-200b were predicted with the help of TargetScan6.2. **(C,D)** Relative luciferase activity as expressed with firefly/renilla luciferase activity. Values are means ± SD (*n* = 5/group). **(C,D)** ^*^P < 0.05 vs. control group; ^#^*P* < 0.05 vs. RhoA wt.pre-miRcon group; ^▵^*P* < 0.05 vs. ROCKII wt.pre-miR-200b con.

## Discussion

The primary goals of this study were to identify the critical miRNAs associated with RMP7-induced increases in BTB permeability and identify some of the underlying mechanisms related with this effect. We took advantage of gene chip technology to detect miRNA profiles in two basic groups—the BTB control and RMP7 treated groups. Microarray, combined with confirmatory quantitative RT-PCR analyses revealed a significant deregulation in miR-200b in the RMP7 group, which led to an increased expression of their target genes, RhoA and ROCK II. MiR-200b directly targeted RhoA and ROCK by binding to specific sites which mediate RMP7-induced changes in actin cytoskeleton rearrangement, TJ-associated protein redistribution and BTB permeability. To our knowledge, this is the first report demonstrating that miRNA is involved in an RMP7-induced increase in BTB permeability.

RETRACTED

Results from preclinical studies have confirmed that RMP7 not only increases BBB, but BTB permeability as well (Prados et al., 2003). Our current *in vitro* results indicate that BTB permeability to RMP7 achieved maximal levels at 15 min, and decreased thereafter. Interestingly, even with a continuous infusion of RMP7, spontaneous barrier restoration was shown to occur within 10–20 min (Bartus et al., 2000; Kraemer et al., 2002); and a rapid, but reversible, and relatively selective permeability of the BTB to RMP7 has also been reported (Packer et al., 2005). As RMP7 has a longer plasma half-life when compared with BK, an exact explanation for the limited duration of BTB permeability to RMP7 is not readily apparent. One possibility is the potential for an auto-regulated internalization of B2 receptors in cells (Pizard et al., 1999).

Microarrays have made rapid progress as a high-throughput screening and high-performance technology. There are miRNAs, specifically miR-181a and miR-34c, that have been reported to be associated with TJ disassembly in the BTB, but not in the BBB (Ma et al., 2014b; Zhao et al., 2015). The miR-34c regulated permeability of the BTB has been shown to result from MAZ-mediated expression changes of ZO-1, occludin and claudin-5 (Zhao et al., 2015). While the miR-181a regulated BTB permeability involves targeting of the Krüppel-like factor 6 (Ma et al., 2014b). These miRNAs expression changes are believed to be associated with deregulation of the target genes which contribute to TJ disassembly and increases in BTB permeability. In our study, use of gene chip technology failed to detect expression changes of miR-181a and miR-34c in GECs of the BTB by RMP7. These results suggest that miR-181a and miR-34c are not involved in mediating RMP7-induced increases in BTB permeability.

The miR-200 family of miRNAs, which includes miR-200c and miR-141 on chromosome 12 and miR-200a/b and miR-429 on chromosome 1, have been extensively studied as related to the epithelial-to-mesenchimal transition (EMT) of cancer cells. The miR-200 family was recently identified as a suppressor of EMT (Park et al., 2008). MiR-200b is down-regulated in glioma tissues and this down-regulation is correlated with a poor prognosis in gliomas (Peng et al., 2013a; Liu et al., 2014). A change (loss or gain) in the miR-200 family of miRNAs is associated with cancer invasion (Magenta et al., 2011). However, little is known about the interrelationships between miR-200s and properties of the endothelium. MiR-200s have been shown to promote endothelial cell apoptosis and senescence and inhibited the capacity for the endothelium to form tumor angiogenesis (Choi et al., 2011; McArthur et al., 2011; Gill et al., 2012; Pecot et al., 2013). These studies suggest that miR-200b might regulate certain functions of endothelial cells. In the present study, we found that RMP7-induced a decrease in miR-200b expression within GECs of the BTB. Similarly, advanced glycation end (AGE) induced down-regulation of miR-200b in HUVEC (Wu et al., 2014) and a down-regulation of miR-200b was observed in the retina in a diabetic rat model (McArthur et al., 2011). In addition, miR-200b expression was depleted within arsenic-transformed human bronchial epithelial cells showing highly migratory and invasive characteristics (Wang et al., 2014b). When collating these findings with our current results it appears that low expressions of miRNA-200b play a key role in a number of physiological and pathological processes.

RETRACTED

Our current data also demonstrate that overexpression of miR-200b could inhibit endothelial leakage and restore normal TEER values in the BTB. Consistent with our results, Wu et al found that miR-200b and miR-200c mimics also inhibited AGE-induced increases in HUVEC permeability (Wu et al., 2014). Moreover, miR-200b mimics prevent glucose-induced increases in permeability and angiogenesis within the retina of diabetic rats (McArthur et al., 2011). Taken together, these results suggest that miR-200b significantly changes the integrity and permeability of the BTB or endothelium.

MiRNAs are small endogenous RNAs that pair with sites in mRNAs to direct post-transcriptional repression. Many sites that have been identified to match the miRNA seed (nucleotides 2–7), particularly those in the 3′-UTR, are preferentially conserved (Friedman et al., 2009). Moreover, the seed pairing site in the 3′-UTR target is often conserved across multiple species (Wang and El Naqa, 2008). MiRNAs can inhibit target gene expression at the post-transcriptional level, which can then play an important role in a wide array of biological processes including embryonic development, cell stress responses and oncogenesis (Keene, 2007; Chang et al., 2013a). Here we provide evidence demonstrating that miR-200b simultaneously regulated the expression of RhoA and ROCKII which results in F-actin rearrangement, relocalization of occludin and claudin-5, TJ opening and increased BTB permeability. Similar results were observed for miR-200b, in that it was also shown to simultaneously regulate ROCKII and SUZ12 gene expression at the post-transcriptional level (Peng et al., 2013b), where ROCKII can participate in the regulation of cytoskeletal signaling events. Recent findings have demonstrated miR-200b results in F-actin rearrangement by directly targeting PKCα (Wang et al., 2014b). It has also been reported that miRNA-200b could promote cell cycle and actin cytoskeletal rearrangement by directly targeting RND3, which was considered to be a natural endogenous antagonist of RhoA (Xia et al., 2010). Accordingly, these studies lend credence to the possibility that miRNA-200b was closely related to molecular events involved with cytoskeletal rearrangement.

RETRACTED

Our results demonstrate that miR-200b directly binds to RhoA and ROCKII 3′-UTR at positions 133–139 and 912–918, respectively. AGE-induced miR-200b and miR-200c down-regulation leads to an increase in the expression of their target genes, RhoA and ROCK II in HUVEC, respectively. Moreover, findings demonstrating that the seed region of miR-200b binds to the RhoA 3′-UTR position are consistent with our findings (Peng et al., 2013b). The miR-200b/c 429 cluster is considered to have the same seed region that binds to the target gene mRNA. The report that the seed region of miR-200c binds to the same RhoA 3′-UTR position in the process of trabecular meshwork cell contraction regulation, is also consistent with our findings (Luna et al., 2012). The seed regions of miR-200b and miR-200c that bind to the RhoA 3′-UTR position in the process of suppressing hepatocellular carcinoma metastasis are also in accordance with our findings, but the seed regions of miR-200b and miR-200c that bind to the ROCKII 3′-UTR position in above-mentioned process were at position 1006-1013, which is inconsistent with our results (Wong et al., 2015). These variations in binding sites to ROCKII may be due to different conservative features located in sites 912-918 and 1006-1013. In addition, it has been demonstrated that MicroRNA-155 contributed to epithelial cell plasticity by targeting RhoA (Kong et al., 2008); and, RhoA had also been confirmed to be a direct target gene for miR-31 during OSCC tumorigenesis (Chang et al., 2013b). The data indicating a discrepancy in the miRNA regulation of RhoA are likely due to differences in treatments factors and/or different protocols.

RETRACTED

## Conclusion

Our results suggest that RMP7 induced miR-200b down-regulation as revealed by microarray and quantitative RT-PCR. MiR-200b directly targeted RhoA and ROCKII, initiating a signaling cascade that resulted in changes of RhoA and ROCKII gene expression, stress fiber formation, TJ protein disassembly and an increase in BTB permeability. The exact mechanism(s) through which RMP7 repressed miR-200b expression as well as an assessment of these effects in *in vivo* models remains to be determined in future studies.

## Author contributions

Conceived and designed the experiments: TM and YX. Performed the experiments: TM. Analyzed the data: TM. Contributed reagents/materials/analysis tools: TM and YX. Wrote the manuscript: TM and YX.

### Conflict of interest statement

The authors declare that the research was conducted in the absence of any commercial or financial relationships that could be construed as a potential conflict of interest.

## Abbreviations

3′-UTR: 3′-untranslated region
AGE: Advanced glycation end
BBB: blood-brain barrier
BK: bradykinin
BTB: blood-tumor barrier
BSA: bovine serum albumin
D-PBS: Dulbecco's phosphate-buffered saline
DMEM: Dulbecco's modified Eagle's medium
ECs: human cerebral microvascular endothelial cells line hCMEC/D3
EDTA: ethylenediamine tetraacetic acid
EMT: epithelial-to-mesenchimal transition
HRP: Horseradish
PAGE: SDS-polyacrylamide gel electrophoresis
miRNAs: MicroRNAs
Quantitative RT-PCR: Reverse Transcription and Quantitative Real Time PCR
SDS: sodium dodecyl sulfate
TEER: transendothelial electric resistance
TJ: tight junction.
